# Hypersensitivity Reaction to a Mosquito Bite in a Patient with Chronic Myeloid Leukemia

**DOI:** 10.1155/2011/649548

**Published:** 2011-10-05

**Authors:** Uri P. Dior, Shaden Salameh, Yonatan Gershinsky, Ruth Stalnikowicz

**Affiliations:** ^1^Department of Emergency Medicine, Hadassah University Hospital, Mount Scopus, P.O. Box 12000, 91120 Jerusalem, Israel; ^2^Department of Internal Medicine, Hadassah University Hospital, Mount Scopus, P.O. Box 12000, 91120 Jerusalem, Israel

## Abstract

A twenty-one-year-old male patient with an exaggerated hypersensitivity reaction to a mosquito bite presented to the department of emergency medicine for further evaluation. He was noted on physical examination to have splenomegaly. The hematological blood tests that were performed were compatible with chronic myeloid leukemia (CML). In this case, the mosquito bite heralded the diagnosis of CML.

## 1. Introduction

Exaggerated reaction to insect bites, mainly to mosquitoes, has been known to be associated with a few hematologic malignancies. This phenomenon has been described mostly in chronic lymphocytic leukemia [1–4] and mantle cell lymphoma [5, 6], but has also been found rarely in acute lymphocytic leukemia, acute monocytic leukemia, and large cell lymphoma [7].

Usually, skin lesions appear months to years after the diagnosis of leukemia has been made and are unrelated to laboratory findings, disease course, or therapy. To the best of our knowledge, we describe the first reported case of exaggerated reaction to insect bite associated with chronic myelogenous leukemia. Furthermore, in this case the exaggerated reaction led to the hematological diagnosis.

## 2. Case Report

A 21-year-old previously healthy male soldier presented to the Department of Emergency Medicine (ED) for evaluation of swelling and pain in both legs. He stated that two evenings earlier, he was stung in both feet by an insect, most likely a mosquito. Immediately after he was stung, he felt an itching sensation, without swelling or pain. The following morning swelling appeared in both of his feet. The patient was referred to a general practitioner who prescribed an antihistamine tablet (chlorpheniramine) and an unknown cream. There was no improvement and antibiotic treatment was prescribed the next day. Despite the antibiotics, the swelling continued to spread, resulting in his decision to present to the ED. On presentation to the ED, he complained of severe itching and pain and swelling spreading from his feet to his legs. He denied chest pain, shortness of breath, abdominal pain, back pain, or headache. He denied having any fever for the previous two days. 

His past medical history was unremarkable. A week before his present admission to the ED, he had complained of left upper quadrant pain. No prior history of allergy or drug sensitivity was reported. The patient's blood pressure was 125/76 mmHg, pulse rate 92 beats/min, respiratory rate 16 breaths/min, temperature 36.5°C (97.1°F), and oxygen saturation 97% on room air. His physical examination was remarkable for pitting edema in his left foot and a mild swelling of his right foot. Diffuse erythemas, as well as localized erythematous papules consistent with insect bites, were observed on both legs. There was no induration or fluctuation suggestive of cellulitis or abscess. One small and tender lymph node was palpated in his left groin. No other enlarged lymph nodes were found. The abdominal examination demonstrated left upper quadrant tenderness and a palpable spleen. The remainder of the physical examination was normal.

Hematologic studies revealed a white blood cell count of 44,300/mm^3^, a platelet count of 164,000/mm^3^, and a hemoglobin level of 14.1 gm/dL. The white blood cell differential revealed 66.5% neutrophils, 25% lymphocytes, 24.6% monocytes, and 2.6% basophiles. Electrolytes, blood urea nitrogen level, glucose and renal function tests were normal. Liver function tests were normal except for a mild elevation of the aspartate aminotransferase (AST) level up to 68 U/L (normal range 2–60 U/L). Lactate dehydrogenase (LDH) was markedly elevated up to 4,513 U/L (normal range 300–620 U/L) and the uric acid was 487 umol/L (150–380 umol/L). Calcium, phosphorus, total protein, albumin, and creatinine kinase levels were normal. 

Twelve hours after presenting to the ED and prior to initiating any treatment, a new rash developed. The rash, involving the neck, upper chest, upper back, and the left forearm was erythrodermic, well demarcated and non-pruritic. This rash resolved spontaneously 12 hours later. 

A peripheral blood smear performed after the initial blood work showed elevated numbers of basophil, blasts, and immature myeloid cells. The patient was transferred from the ED to the hematology department for further evaluation. 

An abdominal ultrasound was performed revealing splenomegaly measuring 17.5 cm with no evidence of infarction. Aspiration and biopsy of the bone marrow were performed. Direct visualization showed hyperplasia of all elements of the granulocyte series. Maturation of the erythroid and granulocytic series was normal. An elevated number of megakaryocytes and eosinophils were noticed and the myeloerythroid ratio was high. Molecular diagnosis revealed 6.25*E*+5 copies per reaction of BCR-ABL with a 94% BCR-ABL to ABL ratio. Further genetic evaluation of the chromosomes derived from the bone marrow sample showed a karyotype with the reciprocal translocation T(9;22) (Q34;Q11) known as the Philadelphia chromosome. The pathologic examination of the biopsy sample demonstrated a significant increase of the myeloid lineage cells, composed mostly from immature eosinophils. The diagnosis of intermediate Sokal score chronic myelogenous leukemia was established.

## 3. Discussion

Chronic myelogenous leukemia (CML) is a hematological stem cell disorder characterized by excessive proliferation of cells of the myeloid lineage. The genetic hallmark of CML is the Philadelphia chromosome, which arises from a reciprocal translocation between chromosomes 9 and 22 that fuse the c-ABL tyrosine kinase gene on chromosome 9 and the breakpoint cluster region (BCR) gene on chromosome 22. The disease is characterized by a chronic phase that can last for months or years and may exhibit few or no symptoms. Eventually, the chronic phase progresses to a more dangerous accelerated or acute (blast crisis) phase, during which the leukemia cells acquire additional genetic changes, proliferate more rapidly, and become resistant to apoptosis, and, if untreated, ultimately cause the patient's demise [8]. In a recent review [9], the median age at the time of diagnosis was 60, and the youngest patient age was 28. Exposure to ionizing radiation is the only known risk factor [10]. The clinical findings at diagnosis of CML vary among reported series and also depend upon the stage of disease at diagnosis. Twenty to 50 percent of patients are asymptomatic, with the disease first being suspected from routine blood tests. Among symptomatic patients, left upper quadrant abdominal pain and early satiety, due to enlargement of the spleen with or without perisplenitis and/or splenic infarction, may occur [11]. Other frequent findings include splenomegaly (present in 48% to 76% in two series), anemia (45% to 62%), white blood cell counts above 100,000/microL (52% to 72%), and platelet counts above 600,000 to 700,000/microL (15% to 34%) [10, 11]. 

A large local reaction to an insect bite is defined as edema and erythema at the site of the bite, with a diameter greater than 10 cm and peaking in intensity at 24–48 hr. It can be evoked by a toxic mechanism, but it is generally believed that an IgE-mediated or even cell-mediated pathogenesis occurs in the majority of cases [12]. The prevalence of large local reactions to insect bites in the general population is variable across studies, and it has been reported to range from 2.4 to 10%, with a maximum of 26.4% [13]. 

The occurrence of unusual hypersensitivity phenomena has been described in patients affected with a few hematologic disorders. The most frequent disorder where this phenomenon has been described is CLL [2, 3]. Weed [2] termed these reactions as an “exaggerated delayed hypersensitivity to mosquito bites”. The hypothesis of an immunoallergic pathway, related to the onset of the cutaneous eruption, has been proposed [14]. 

In our emergency department, blood tests are not routinely drawn in patients with a presumed diagnosis of allergic reaction. However, the finding of splenomegaly and left upper quadrant tenderness raised the suspicion of an underlying disease. 

The diagnosis of CML is very rare at this young age, and hypersensitivity response to insect bite in CML has not been previously reported. This combination seems unique, and we suggest that when an exaggerated response to insect bite is encountered, further investigation for potential underlying disease is recommended.
